RETRACTED

# A Blumgart Anastomosis-Based Half-Invagination Pancreaticoenterostomy with Better Applicability to Laparoscopy and Lower Incidence of Pancreatic Leakage

**DOI:** 10.1155/2023/6304047

**Published:** 2023-02-23

**Authors:** Qiang Sun, Peng Peng, Xueyi Gong, Jianlong Wu, Qiao Zhang, Zhipeng Hu, Xiaojian Chang, Zemin Hu

**Affiliations:** General Surgery Department 1, Zhongshan People's Hospital, Zhongshan Hospital Affiliated to Sun Yat-Sen University, Zhongshan, China

## Abstract

**Background:**

The Blumgart anastomosis (BA) is one of the safest anastomoses for pancreatic stump reconstruction. The incidence of postoperative pancreatic fistula (POPF) and postoperative complications is low. However, how to make laparoscopic pancreaticoenterostomy easier and safer is still a topic to be discussed.

**Methods:**

The data of patients who underwent laparoscopic pancreaticoduodenectomy (PD) from April 2014 to December 2019 were analyzed retrospectively.

**Results:**

Half-invagination anastomosis was performed in 20 cases (HI group), and the Cattell-Warren anastomosis was carried out in 26 cases (CW group). The amount of intraoperative bleeding, operation time, and postoperative catheterization time in the HI group was significantly less than those in the CW group. Besides, the number of patients at the Clavien-Dindo grade III and above in the HI group was significantly less than that in the control group. Moreover, the incidence of POPF in the HI group was significantly lower than that in the CW group. Furthermore, fistula risk score (FRS) analysis showed that there was no high-risk group, and the highest risk in the medium-risk group was pancreatic leakage. In addition, the incidence of pancreatic leakage in the HI group and CW group was 7.7% and 46.67%, respectively, while the incidence of pancreatic leakage in the HI group was significantly lower than that in the CW group.

**Conclusions:**

The half-invagination pancreaticoenterostomy based on the Blumgart anastomosis should have good applicability under laparoscopy and could effectively reduce the incidence of postoperative pancreatic leakage.

## 1. Introduction

Since Gagner and Pomp reported the first case of complete laparoscopic pancreaticoduodenectomy (LPD) in 1994, it has been developed very rapidly. Especially in the past 10 years, LPD has become a routine operation in numerous pancreatic centers [1]. There are obvious advantages of LPD for hospital stay and intraoperative blood loss, as its short-term or long-term efficacy is similar or even better than that of open pancreaticoduodenectomy (OPD) [2–6]. However, some studies are against LPD [7, 8], because LPD is one of the most complex laparoscopic surgery and required higher techniques and longer learning curve [2]. As with laparotomy, the quality of pancreaticointestinal anastomosis is still the key factor for postoperative complications and mortality. There are many methods utilized for pancreaticointestinal anastomosis, including duct-to-mucosa pancreaticojejunostomy (PJ), end-to-side PJ, binding PJ, invagination PJ, and pancreaticogastrostomy. Nevertheless, there is no effective method to reduce the incidence of pancreatic leakage [9]. In 2000, Professor Blumgart introduced a pancreaticointestinal anastomosis with U-shaped suture called the Blumgart anastomosis, which can significantly reduce the occurrence of postoperative pancreatic leakage [10]. In 2009, Kleespies et al. and Grobmyer et al. reported the detailed methods and effects of the Blumgart anastomosis [11, 12]. Since then, many improved methods have been reported. It has been indicated that the incidence of pancreatic leakage in the Blumgart anastomosis is 2.5%-20.5%, which is lower than that in the Cattell-Warren anastomosis, Kakita anastomosis, and pancreatogastric anastomosis [13–21].

RETRACTED

Despite the rapid development of laparoscopic instruments and surgical techniques, it is unclear whether laparoscopy can be successfully applied to laparoscopic surgery due to the different operating characteristics of laparoscopy and laparotomy [22]. How to make laparoscopic pancreaticoenterostomy easier and safer to promote the wider and more standardized implementation of LPD is still a topic to be discussed [22]. At present, laparoscopic pancreaticoenterostomy mainly adopts pancreatic duct mucosal anastomosis and end-to-side anastomosis, most of which are the same as laparotomy [22]. In addition, some surgeons have improved the characteristics of laparoscopy and achieved promising results [23–26].

The Blumgart anastomosis is a kind of pancreatic duct mucosal anastomosis, which is mainly used for laparotomy. However, the Blumgart anastomosis is rarely used for laparoscopic surgery [27, 28]. This study reported a modified Blumgart pancreaticointestinal anastomosis based on the characteristics of laparoscopy and compared it with the laparoscopic Cattell-Warren pancreaticointestinal anastomosis for the first time. A preprint of the current study has previously been published in Research Square [29].

## 2. Materials and Methods

### 2.1. Patients

46 patients who underwent laparoscopic pancreaticoduodenectomy (PD) in Zhongshan People's Hospital from April 2014 to December 2019 were recruited in this study. All cases were performed by two groups of doctors. The two groups of doctors have similar skilled and stable experience in open pancreaticoduodenectomy. Dr. Xiaojian Chang's team has used the modified Blumgart half-invagination pancreaticoenterostomy (HI group) since May 2017, while Dr. Zemin Hu's team has always used the Cattell-Warren anastomosis (CW group). Of the 46 patients retrospectively analyzed in this study, 31 were completed by Dr. Xiaojian Chang's team (20 cases of HI method and 11 cases of CW method), and 15 cases (CW method) were completed by Dr. Zemin Hu's team. Informed consent was obtained from all individual participants included in the study. All procedures in the present study were performed in Zhongshan Hospital Affiliated to Sun Yat-Sen University with the approval of the Ethics Committee. All methods were performed in accordance with all relevant guidelines and regulations.

RETRACTED

### 2.2. Surgical Procedure

LPD was performed on the patient lying on his back, with his legs separated and in a slight anti-Trendelenburg position. A holder of the mirror stood between the legs, with an operator and an assistant on either side of the patient. A total of 5 trocars were placed. Three trocars with a diameter of 12 mm were located about 5 cm below the umbilicus and on the left and right sides of the umbilicus, respectively. Two 5 mm trocars were placed in the left and right epigastrium. Except 2 cases with Olympus 3D laparoscopy, the rest were performed with 30° 2D laparoscopy.

All cases underwent partial distal gastrectomy without preserving pylorus. Patients with malignant tumors underwent lymph node dissection, including duodenal ligament, common perihepatic artery, peripancreatic head, celiac trunk, and left superior mesenteric artery lymph nodes. Concomitant portal vein and/or superior mesenteric vein (PV/SMV) resection is performed on patients with possible or definite tumor invasion. The reconstruction process was carried out by a “CHILD” method. The upper intestinal segment was lifted to the subhepatic portion through the mesenteric root. First, pancreaticoenterostomy was performed at about 5 cm away from the ruptured end of the jejunum. Second, choledochojejunostomy was performed at about 5-15 m away from the position of pancreaticoenterostomy. When the diameter of bile duct was ≥1.0 cm, 4-0 V-Loc was used for end-to-end anastomosis of bile duct and jejunum; when the diameter of the bile duct was less than 1.0 cm, 4-0 Monocryl suture was used for intermittent suture and placed internal stents. Finally, the gastrojejunal side-to-side anastomosis was performed before the colon. A drainage tube was placed in front of and behind the pancreaticoenterostomy site.

### 2.3. Cattell-Warren Pancreaticoenterostomy

The dorsal muscle layer and jejunal muscle layer of pancreatic stump were sutured with 3-0 Prolene suture. A small incision was made at the corresponding jejunum to mesentery for the anastomosis of pancreatic duct to mucous membrane. Pancreaticostomy was a continuous suture with 5-0 Prolene suture after placing a suitable sten. If the diameter of the pancreatic duct was ≤3 mm, suture was carried out intermittently. Finally, the same method was used to complete the anastomosis between the ventral side of the pancreatic stump and the seromuscular layer of the jejunum.

RETRACTED

### 2.4. Half-Invagination Pancreaticoenterostomy

U-shaped suture was performed with 3-0 or 4-0 Prolene suture according to the thickness of pancreatic stump. Double needle Prolene suture was cut into 15 cm, and the tail knot was tied for standby (3 in total). Steps of half-invagination pancreaticoenterostomy were listed as follow: step 1: suture A: the sarcoplasmic layer was sutured from top to bottom parallel to the long axis of the jejunum about 1 cm away from the pancreatic stump and inserted from the posterior wall. Then, the pancreatic parenchyma was sutured in full layer. The other needle was perpendicular to the long axis of the jejunum and sutured with sarcoplasmic muscle layer, about 1 cm away from the pancreatic stump. The whole layer of the pancreatic parenchyma was sutured at the upper edge of the pancreas (Figures 1(a) and 1(b)). Next, the suture was tightened so that the pancreatic stump was closed to the jejunum and fixed with a vascular clamp (the suture is not knotted) to facilitate tension-free anastomosis between the pancreatic duct and the mucosa (Figures 1(c) and 1(d)). Step 2: suture B: two needles parallel to the long axis of the jejunum were used to suture the sarcoplasmic layer of the jejunum, which was inserted through the posterior wall about 1 cm away from the pancreatic stump of the head and tail of pancreatic duct. The pancreatic parenchyma was sutured in full thickness without knots (Figures 1(c) and 1(d)). Step 3: after placing the appropriate pancreatic duct stent, the anastomosis between pancreatic duct and mucosa was continuously sutured with 5-0 Prolene suture. The diameter of pancreatic duct was less than 3 mm, and then, intermittent suture was carried out. Step 4: suture C was used to suture symmetrically with the first suture. Henceforth, the jejunum was inserted into the back of the pancreatic stump (Figures 1(e) and 1(f)). Step 5: from the tail to the head, the endoplasmic muscle layer was sutured symmetrically with the dorsal side of the pancreatic stump with C followed by B and A sutures (Figures 1(g) and 1(h)). The suture position was about 1-1.5 cm away from the jejunum corresponding to the pancreatic stump and knot them separately (Figures 1(i) and 1(j)) to complete the ventral insertion of the pancreatic stump (Figures 1(k) and 1(l)).

RETRACTED

### 2.5. Perioperative Management and Definition of Postoperative Complications

If the patient's preoperative total bilirubin was >300 mmol/L, percutaneous transhepatic cholangial drainage (PTCD) should be performed for two weeks to reduce jaundice or preoperative total bilirubin to <51 mmol/L. On the 3rd day after operation, when the flow of nasogastric tube was less than 200 mL/D, nasogastric tube was removed. On the 3rd day after operation, the drainage fluid of abdominal drainage tube was collected, and the concentration of amylase was detected. When the drainage volume was less than 20 mL, drainage tube was removed. On the 5th day after operation, routine computed tomography (CT) scanning was performed on the upper abdomen to understand abdominal abscess and effusion. On the 3rd day after operation, patients began to eat liquid food. All patients were treated with somatostatin analogues.

International Study Group of Pancreatic Surgery (ISGPF) classification was used for the definition of postoperative complications (POPF, delayed gastric emptying, and postpancreatectomy hemorrhage (PPH)) [30–32], while POPF grades B and C were regarded as clinically relevant. Postoperative bleeding was defined as a PPH grade B or C according to the ISGPF [32]. Acute pancreatitis was chemically defined as an elevated serum amylase and/or lipase level (at least three times of the normal level) for at least 3 consecutive days on the 3rd day after operation. Acute pancreatitis was confirmed by CT. The classification of postoperative complications was the Clavien-Dindo classification [33]. The FRS is a 10-point scale that relies on weighted effect of four variables including gland texture, pathology, duct size, and estimated blood loss [34, 35]. The weighted aggregate of these risk factors was used to calculate the individual FRS score (0-10) for each patient.

### 2.6. Statistical Analysis

Continuous data were presented as mean ± standard deviation (SD) or the median (25th-75th percentile) and the difference in statistics analyzed by the Student *t*-test or the Kruskal-Wallis test. The categorical variables were compared by Chi square test and Fisher's exact test and expressed as numbers (percentages). *P* < 0.05 was considered statistically significant. All statistical analyses were performed using SPSS statistical analysis software package v. 19 (IBM SPSS Statistics, USA).

## 3. Results

In this study, 20 patients were enrolled in the HI group and 26 patients were recruited in the CW group. The clinical and statistical characteristics of patients involved in these two groups are shown in Table 1. Except for diagnosis, there was no significant difference in preoperative clinical and statistical characteristics between patients of these two groups. The number of cases of periampullary carcinoma was higher in the CW group. The intraoperative bleeding (50.00 (45.00, 162.50) vs. 125.00 (100.00, 287.50), *P* = 0.008) and operation time (352.5 ± 99.55 vs. 426.5 ± 106.47, *P* = 0.020) in the HI group were significantly lower than those in the CW group. There was no significant difference in pancreatic texture between two groups. The time of placing PJ drainage tube in the HI group was significantly shorter than that in the CW group (11.00 (10.00, 13.50) vs. 12.50 (11.00, 19.00), *P* = 0.009). The diameter of pancreatic duct in the HI group was significantly lower than that in the CW group (3.00 (2.00, 3.25) vs. 4.00 (3.00, 5.00), *P* = 0.013), and the number of pancreatic ducts with diameter ≤ 3 mm in the HI group was significantly higher than that in the CW group (15 vs. 11, *P* = 0.038). In addition, there was no significant difference in postoperative hospital stay between two groups.

RETRACTED

Besides, the postoperative complications are shown in Table 2. The incidence of postoperative complications was similar between two groups, whereas the incidence of patients at the Clavien-Dindo grade III or above in the HI group was significantly lower than that in the control group (2 vs. 10, *P* = 0.043). The incidence of POPF was 5% and 34.6% in the HI group and CW group, respectively (*P* = 0.028). On the 3rd day after operation, the amylase of drainage fluid in the HI group was dramatically lower than that in the CW group (214.50 (77.25, 817.25) vs. 1418.00 (408.75, 3674.50), *P* = 0.020). Unfortunately, one patient died in each group. The patient of the HI group died of unrelated postoperative pulmonary embolism complications, while the patient of the CW group died of abdominal bleeding, abdominal infection, and leakage caused by multiple organ failure. According to the analysis of fistula risk score (FRS), the incidence of pancreatic leakage at different level was different. Due to the significant reduction in bleeding after laparoscopic surgery, there was no high-risk patient in this study, while the highest risk in the medium-risk group was pancreatic leakage. The incidence of pancreatic leakage in the HI group and CW group was 1/13 (7.7%) and 7/15 (46.67%), respectively, and the incidence rate of group HI was significantly lower than that of group CW (*P* = 0.038).

## 4. Discussion

In an open surgical environment, clinical evidence suggests that there is no better surgical option for the reconstruction of residual pancreas except PD, which may depend on the surgeon's expertise, experience, the texture of the pancreas, and the patient's condition [22, 36, 37]. To date, we should pay attention to the following four points in PD: pancreatic juice should be completely drained, blood flow should be maintained at the pancreatic stump, pancreatic parenchyma tear should be prevented, and the jejunal wall should be in close contact with pancreatic section [38]. In order to meet the surgical characteristics of laparoscopic pancreaticoenterostomy, the following points should also be considered: (1) is it simple? (2) Is it technically easy and feasible? (3) Is it safe? (4) Is there any scientific evidence to support it [22]?

RETRACTED

In this study, there were more cases of thinner pancreatic ducts with diameter ≤ 3 mm in the HI group, which may be related to the different diagnosis of two groups. Studies have shown that diameter of pancreatic duct ≤ 3 mm is an independent risk factor for pancreatic leakage [39]. Nevertheless, the incidence of pancreatic leakage in the HI group was lower than that in the CW group, and the time of postoperative drainage tube placement was shorter. There was no significant difference in postoperative hospital stay between two groups, which may be related to the delayed gastric emptying of 3 patients in the HI group, which significantly prolonged the postoperative hospital stay. Callery et al. and Miller et al. proposed a FRS including four factors: gland texture, pathology, duct size, and estimated blood loss [34, 35]. Accordingly, the factors of pancreatic leakage analysis were analyzed in this study, and results found that the higher the score, the higher the risk of pancreatic leakage. The intermediate risk group had the highest risk of pancreatic leakage, and the incidence of the HI group was significantly lower than that of the CW group. It was worth mentioning that FRS is a risk assessment method of pancreatic leakage based on laparotomy analysis, one of which is intraoperative bleeding. Previous studies have shown that laparoscopic surgery can significantly reduce intraoperative blood loss. Therefore, FRS could not fully reflect the characteristics of laparoscopic surgery and may need to be adjusted.

The methods used in this study have been previously reported in laparotomy [17]. According to the characteristics of laparoscopic surgery, we improved this method and considered that it might be more suitable for laparoscopic surgery.

The hemostatic methods of open and laparoscopic pancreatic sections are different. In laparotomy, small blood vessels and pancreatic ducts can be carefully dissected and ligated, but under laparoscopy, ultrasonic scalpel and electrocoagulation are usually used, which usually lead to eschar shedding, bleeding, or trace pancreatic leakage. U-shaped suture is conducive to hemostasis of pancreatic stump and reduces pancreatic leakage of small pancreatic duct. Therefore, it is recommended to use the Blumgart method based on U-shaped suture under laparoscopy. The traditional Blumgart method requires 4-6 U-shaped sutures [12], and too many sutures are not conducive to laparoscopic surgery. Compared with the traditional Blumgart method, the method mentioned in this study can reduce the number of stitches of U-shaped sutures, facilitate laparoscopic suture, reduce the bleeding of pancreatic stump, and preserve the blood supply of the pancreatic stump as much as possible. Scissors are often used to cut off the main pancreatic duct. However, there are blood vessels near the main pancreatic duct. Therefore, the second U-shaped suture is helpful to reduce the bleeding of the pancreatic sections and the effusion between the jejunum and the pancreatic section [38, 40].

RETRACTED

In order to make the jejunum better cover the pancreatic stump, we optimized the “U” suture method of the upper and lower edges of the pancreas to make the jejunum better adapt to the pancreatic stump (as shown in Figure 1). In this study, pancreatic duct stents were placed in all cases, which had not been described in the traditional Blumgart method [11]. Although it is not clear whether stent could reduce pancreatic leakage [41], the placement of the stent after the suture of the posterior wall of pancreatic duct is conducive to the suture of the anterior wall. In addition, we still believed that the second “U” suture combined with the pancreatic stent could reduce the risk of pancreatic fluid leakage to mucosal anastomosis site through the pancreatic duct.

In our method, all the knots were on the serosa surface of the jejunum. The pancreatic parenchyma was unknotted, which could withstand greater tension because the pancreatic parenchyma had no cutting force. Even if there was anastomotic edema after operation, the tissue cutting can be reduced as much as possible. Although laparoscopic suture tension is more difficult to master than laparotomy, the above suture method can reduce the difficulty of laparoscopic suture, shorten the learning curve, and improve the safety of pancreaticointestinal anastomosis. When the pancreatic duct is located at the posterior edge of the pancreas and anastomosed by the Kakita and Cattell-Warren methods, the needle eye of anastomosis between the posterior wall of the pancreatic duct and the jejunum is not easy to be covered by the jejunum, resulting in pancreatic leakage. In our method, all needles of pancreatic parenchyma were covered by the jejunum, which reduced the occurrence of pancreatic leakage. Oh first reported the shortcomings of the modified Blumgart method [20]. When the jejunal tube is small in diameter and increased or thickened relative to the pancreatic stump, the jejunal insertion may be incomplete, resulting in a shear force parallel to the long axis of the pancreas and tearing of the pancreaticojejunal anastomosis [20]. Our experience for practical application was consistent. Therefore, we believed that the sarcoplasmic suture along the long axis of the jejunum [11, 15, 17] made it easier for the jejunum to insert into the pancreatic stump than along the short axis of the jejunum [12, 14, 38], and the stress range was larger, and the cutting was more difficult, especially when pancreatic stump is thicker or the jejunum is thinner [20].

RETRACTED

At present, the laparoscopic Blumgart pancreaticoenterostomy is rare [27, 28]. Poves et al. first reported the modified laparoscopic Blumgart pancreaticoenterostomy. In addition, the modified laparotomy Blumgart pancreaticoenterostomy is used for paired comparison. In the laparoscopic group, the incidence of postoperative Clavien grade III or higher complications and hospital stay is reduced. When implementing this method, an additional 5 mm trocar is inserted into the upper abdomen in front of the planned PJ. Through this trocar, the 2-needle polypropylene 2–0 MH 36 mm 1/2 c 90 cm transpancreatic stitches are externalized [27]. Then, the pancreatic stump moved at least 3 cm from the edge of the pancreas section. Our method could shorten the length of suture and facilitate laparoscopic surgery. The first suture was fixed with vascular clamp, and the jejunum was close to the pancreatic stump, so that the anastomosis between the pancreatic duct and mucosa could be completed without tension. At the same time, it avoided pulling the suture out of the body through another trocar, which was convenient for operation.

Peng et al.'s binding pancreaticoenterostomy inserts the pancreatic stump into the jejunum to suture the pancreatic stump and jejunum, which does not penetrate the jejunal muscle layer [42, 43]. After insertion into the jejunum cavity, pancreatic stump is bound around the jejunum and pancreas, and the two are bound together to avoid pinholes on the surface of the pancreas, so as to significantly reduce the incidence of pancreatic leakage. Peng et al.'s binding pancreaticoenterostomy is a nested method. There is no residual pinhole in pancreas by binding, thereby reducing pancreatic leakage. In the study performed by Maggiori et al., the fistula rate of traditional PJ and binding technique are similar, but the fistula healing time of PJ patients using Peng et al.'s technique is longer than that of traditional PJ (29 days and 9 days, respectively) [44]. The incidence of bleeding is also higher in the binding technique (6/22 vs. 0/25). The method used in the current study, through U-shaped suture and half invagination of the jejunum, not only led to hemostasis and reduced anastomotic bleeding but also resulted in pancreatic stump and half invagination of the jejunum on the needle hole on the surface of pancreas. Therefore, we called it half-invagination pancreatic duct mucosa anastomosis.

RETRACTED

However, it has also been reported that the incidence of pancreatic leakage of the modified Blumgart method is consistent with that of the Cattell-Warren method and Kakita method [45, 46]. Kawakatsu et al. reported the application of this technique in soft pancreas [45]. The incidence of pancreatic leakage by the above method and Kakita method is 42.7% and 42.6%, respectively, with no significant difference. Lee and Kim compared the Blumgart method and Cattell-Warren method and found that the incidence of pancreatic leakage is 13.7% and 2.3%, respectively [46]. However, these results may need to verify by more cases. Recently, Hirono et al. reported a prospective randomized controlled study that improved the Blumgart and Kakita methods [38]. The incidence of pancreatic leakage in the two groups is 10.3% and 6.8%, respectively. The incidence of complications is also similar between two groups.

There were still some limitations in this study. First, this study was a retrospective study with only a small size of cases. Besides, the cases in the CW group were completed by two groups of doctors, which may lead to bias in case selection and surgical skills. Moreover, we compared the effects of two laparoscopic pancreaticojejunostomies for the first time. In addition, randomized controlled trials (RCTs) should be needed to assess the real value of laparoscopic approach in PD.

## 5. Conclusion

In conclusion, the method proposed in this study could effectively reduce the incidence of postoperative pancreatic leakage and serious complications. This method should be a more convenient, easier, and safer half-invagination pancreatic duct to mucosal anastomosis and more suitable for laparoscopic surgery.

## Figures and Tables

**Figure 1:** Half-invagination pancreaticoenterostomy. (a, b) Suture A: the two needles were sutured perpendicular to the long axis of the jejunum to the sarcoplasmic muscularis, about 1 cm away from the pancreatic stump, and the full-thickness of the pancreas parenchyma. (c, d) Fixed the suture A with vascular clamp (the suture is not knotted), so as to facilitate the anastomosis of pancreatic duct to mucosa without tension; suture B: two needles were parallel to the long axis of the jejunum to suture jejunum sarcoplasmic layer and then were inserted from the head side and tail side of pancreatic duct through paries posterior about 1 cm from the pancreatic stump. The pancreatic parenchyma was sutured in full thickness without knots. (e, f) Pancreatic duct to the mucosa anastomosis was performed after appropriate pancreatic duct stent tubes were placed. Used suture C to suture symmetrically with the suture A. (g, h) From the tail to the head, C, B, and A sutures were sequentially used to suture the jejunoplasmic muscle layer in a symmetrical manner with the dorsal side of the pancreatic stump and knot separately. (i, j) Completed the insertion of the ventral side of the pancreatic stump. (k) Side view post suture. (l) Dorsal side of the pancreaticointestinal anastomosis, the jejunal serosal layer was inserted into the pancreatic stump.

RETRACTED

**Table 1:** Patient characteristics.

	HI group	CW group	*P*
*N*	20	26	
Age (years)	59.00 (55.50, 65.25)	59.50 (49.50, 65.75)	0.938
Sex ratio (M : F)	12 : 8	11 : 15	0.373
ASA			0.842
Level II	13	15	
Level III	7	11	
Cardiopulmonary disease	5 (25%)	7 (26.9%)	1.000
Diabetes	4 (20%)	4 (15.4%)	1.000
BMI (kg/m^2^)	21.42 ± 3.11	22.38 ± 2.97	0.300
Diagnosis			0.049
Pancreatic cancer	5	5	
Ampullary cancer	3	14	
Bile duct cancer	6	4	
Other	6	3	
Pancreatitis	4	5	1.000
Preoperative biliary drainage	2	3	1.000
Estimated blood loss (mL)	50.00 (45.00, 162.50)	125.00 (100.00, 287.50)	0.008
Transfusion	0	15.38 ± 54.35	0.213
Duration of operation (min)	352.5 ± 99.55	426.5 ± 106.47	0.020
Portal vein resection	1	0	0.435
Duration of PJ drainage tube placement (days)	11.00 (10.00, 13.50)	12.50 (11.00, 19.00)	0.009
Soft/firm pancreas	11/9	11/15	0.552
Pancreatic duct diameter (mm)	2.96 ± 1.40	4.15 ± 1.64	0.0145
≤3 mm (*n*)	15	11	0.038
Postoperative hospital stay (days)	15.50 (12.50, 23.00)	19.50 (13.50, 24.50)	0.417

ASA: American Society of Anesthesiologists; BMI: body mass index; PJ: pancreaticojejunostomy.

**Table 2:** Postoperative complications.

	HI group	CW group	*P*
Total complications (*n*, %)	10 (50%)	16 (61.5%)	0.111
Clavien I-II	8	6	0.333
Clavien III-IV	1	9	0.028
Clavien V	1	1	1.000
Clavien ≥ III	2	10	0.043
Surgery complication			
POPF (B+C)	1 (5%)	9 (34.6%)	0.028
Grade B	1	4	0.369
Grade C	0	5	0.070
Drain AMY level (POD3)	214.50 (77.25, 817.25)	1418.00 (408.75, 3674.50)	0.020
Biliary leakage	0	0	
Postpancreaticoduodenectomy hemorrhage (B+C)	0	5	0.059
Delayed gastric emptying (B+C)	3	0	0.075
Acute pancreatitis	1	2	1.000
Intra-abdominal infection	3	10	0.106
Wound infection	0	1	1.000
Reoperation	0	5	0.059
Nonsurgical complications			
Respiratory events	1	4	0.369
Cardiac events	0	0	
MODS	1	1	1.000
Mortality 90 days	1	1	1.000
Fistula risk score (POPF, %)			0.702
Negligible risk (0)	2 (0)	5 (0)	
Low risk [1, 2]	5 (0)	6 (2, 33.33%)	0.467
Intermediate risk [3–6]	13 (1, 7.7%)	15 (7, 46.67%)	0.038
High risk [7–10]	0	0	

POPF: postoperative pancreatic fistula; AMY: amylase; MODS: multiple organ dysfunction syndrome.

RETRACTED

## Data Availability

The data used to support the findings of this study are included within the article.
